The article "Long Noncoding RNA-EBIC Promotes Tumor Cell Invasion by Binding to EZH2 and Repressing E-Cadherin in Cervical Cancer" was retracted in 2025. Reasons: errors in the methods; duplicated images; duplicated data; unreliable results or conclusions.

# Long Noncoding RNA-EBIC Promotes Tumor Cell Invasion by Binding to EZH2 and Repressing E-Cadherin in Cervical Cancer

**DOI:** 10.1371/journal.pone.0100340

**Published:** 2014-07-09

**Authors:** Ning-xia Sun, Chen Ye, Qian Zhao, Qing Zhang, Chen Xu, Shao-bing Wang, Zhi-jun Jin, Shu-han Sun, Fang Wang, Wen Li

**Affiliations:** 1 Department of Obstetrics and Gynaecology, Shanghai Changzheng Hospital, Second Military Medical University, Shanghai, China; 2 Department of Medical Genetics, Second Military Medical University, Shanghai, China; CSIR Institute of Genomics and Integrative Biology, India

## Abstract

In recent years, long noncoding RNAs (lncRNAs) have been demonstrated to play key roles in tumorgenesis. However, the contributions of lncRNAs to cervical cancer (CC) remain largely unknown. In this study, differentially expressed lncRNAs and mRNAs in cervical cancer and paired peritumoral tissues were detected by transcriptome microarray analysis. We found 708 probe sets of lncRNAs increased and 836 probe sets decreased in CC tissues, while 1288 mRNA differential probe sets increased and 901 mRNA probe sets decreased. The results were validated by quantitative real-time polymerase chain reaction (qPCR). Then, we found a specific differentially expressed lncRNA can physically bind to enhancer of zeste homolog2 (EZH2) by using RNA immunoprecipitation. We termed it as EZH2-binding lncRNA in cervical cancer [lncRNA-EBIC]. Wound healing assays and Matrigel invasion assays were used to determine the function of this lncRNA by silencing it. We observed that the migration and invasion of cervical cancer cells *in vitro* were inhibited upon suppression of lncRNA-EBIC by siRNA. We also found that the association between lncRNA-EBIC and EZH2 was required for the repression of E-cadherin, which was a key molecular in the metastasis of cervical cancer.

**Conclusion:**

These results demonstrated that lncRNA-EBIC was an oncogenic lncRNA, which could promote tumor cell invasion in CC by binding to EZH2 and inhibiting E-cadherin expression.

## Introduction

Cervical cancer (CC) is the second most commonly diagnosed cancer and the third leading cause of cancer death in women [1]. Approximately 49,000 new cases of CC were diagnosed and 275,000 women were killed in 2011, which most occurred in developing countries [2], [3]. In addition to the pathogenesis of persistent, high-risk human papillomavirus (HPV) infections, the contributions of other factors to the development and progression of this malignancy need to be elucidated.

More recently, emerging evidences have demonstrated that epigenetic mechanisms may be the key to initiating tumorigenesis. Disruption of epigenetic control of DNA methylation, RNA regulation, and histone modification, etc, resulting in the heritable variation of genes without a change in their coding sequence, is pervasive in malignancy [4], [5]. Although researches of small noncoding RNAs have dominated the field of RNA regulation in recent years [6], [7], a wide array of cellular functions has also been associated with some newly described classes of noncoding RNAs. One such class, long noncoding RNAs (lncRNAs), is transcript of more than 200 nucleotides with no protein-coding potential. Numerous reports have demonstrated that its misregulation has a functional role in various types of cancers [8]. For instance, lncRNA-HEIH plays a key role in cell cycle regulation of hepatocellular carcinoma cells, and high lncRNA-HEIH expression correlates with an increased risk of recurrence and reduced overall postoperative survival rate [9]. As lncRNAs are emerging as critical components of the cancer transcriptome, it is reasonable to anticipate that lncRNAs contribute to the development and progression of cervical cancer. However, studies on the role of lncRNAs in CC are very preliminary. Until now only one research has detected increased levels of aberrant lncRNA expression in cervical intraepithelial neoplasia (CIN) specimens representing mild, moderate, and severe histopathologic grades, respectively, suggesting that lncRNAs may play important roles in the development and progression of precancerous lesions or carcinomas [10]. However, the overall pathophysiological contributions of lncRNAs in CC remain largely unknown.

A recent study has reported that one-fifth of all human lncRNAs identified to date is physically associated with polycomb repressive complex 2 (PRC2, comprised of histone H3 lysine 27 methylase EZH2, SUZ12 and EED), suggesting that they may have a general role in recruiting polycomb-group proteins to their target genes and leading to transcriptional repression [11]. EZH2 (Enhancer of Zeste Homolog 2) is an critical component of PRC2, which is involved in several important regulatory mechanisms such as stem cell differentiation, cell proliferation, cell cycle, and oncogenesis [12], [13]. There are increasing evidences that EZH2 is often over-expressed in many kinds of human cancers and could promote cell proliferation, invasion, and tumor angiogenesis [14]–[16]. Moreover, several lncRNAs, such as lncRNA-HEIH, H19 and HOTAIR, have been shown to physically bind to EZH2 and play important roles in modulating the cancer epigenome [9], [17], [18]. Based on these findings, we hypothesized that some lncRNAs may also play active roles in the malignant biological behaviors of CC by mediating and cooperating with EZH2.

So it will be interesting to determine the biological functions of lncRNAs in CC and whether they function to recruit PcG proteins to target genes. In this study, through transcriptome microarray analysis, we found a number of lncRNAs up- or down-regulated in CC compared with paired peritumoral tissues. We further identified a new lncRNA which was up-regulated in CC and could physically bind to EZH2 and participate in the regulation of migration and invasion of CC cell lines.

## Materials and Methods

### Ethics statement

The study was approved by the Specialty Committee on Ethics of Biomedicine Research of the Second Military Medical University. Written informed consent was obtained from patients for the use of their tissue samples in this research project.

### Patient characteristics and tissue specimens

Twenty-eight pairs of snap-frozen CC and paired peritumoral tissues were obtained from Shanghai Changzheng Hospital with informed consent and approval by the institutional ethics committee. Clinical tissue samples were verified as tumor or non-tumor by histopathological examination and stored at −80°C until use. The patients' characteristics are detailed in Table S1.

### Microarray and computational analysis

Briefly, five CC tissues and five paired peritumoral tissues (Table S1) were used to synthesize double-stranded complementary DNA (cDNA) by reverse-transcription polymerase chain reaction. Double-stranded cDNA was hybridized to Glue Grant Human Transcriptome arrays (Affymetrix, USA) according to manufacturer's protocol, and Affymetrix® Expression Console Software (version 1.3.1) was used for microarray analysis. Raw data (CEL files) were normalized at the transcript level using the robust multi-average method (RMA workflow). Median summarization of transcript expression was calculated. Gene-level data represented genes found in the Rfamdb, fRNAdb, Ensembl, Noncodedb, and RefSeq databases. Using the same method, exon-level data represented full-length transcripts. The random variance model (RVM) t-test was used to identify differentially expressed genes between the CC and peritumoral groups, without increasing the rate of false positives [19]. We selected differentially expressed genes according to RVM and false discovery rate (FDR) analyses, with a predefined P-value threshold of <0.05 [20]. Hierarchical clustering (Cluster3.0) and TreeView analysis (Stanford University, USA) were performed based on the results of differentially expressed genes. The microarray data discussed in this article have been submitted to National Center for Biotechnology Information (NCBI) Gene Expression Omnibus (GEO) and are accessible through (GEO) Series accession number GSE55940 (http://www.ncbi.nlm.nih.gov/geo/query/acc.cgi?acc=GSE55940).

### Data filtering and establishment of a gene co-expression network

A query design of Microsoft Office Access 2013 was used to overlap differentially expressed genes with the Cervical Cancer Gene Database (CCDB) by gene symbol. Co-expression network analysis was carried out between the genes of overlap and differential lncRNAs to identify gene interactions [21]. Co-expression networks were built according to the normalized signal intensity of specific expressed genes. Firstly, we constructed the network adjacency matrix as previously described [22]. Secondly, we calculated the Pearson correlation for each pair of genes and chose the prominent correlation pairs to construct the network. To make a visual representation, only those genes with the strongest interaction (0.865 or greater) were selected. In the network analysis, a degree is the most important parameter of the centrality of a gene within a network that determines the relative importance. Degree centrality is defined as the number of links one node has to another. To explore the degree difference of certain hub genes and neighbors between cancer and peritumoral groups, |diffK| was introduced to the analysis. The |diffK| is equal to the difference in the standardized degrees of hub genes in 2 groups and suggests that the hub gene may have a stronger ability of regulation in the cancerous or peritumoral region.

### Cell culture

Human cervical cancer cell lines (HeLa, SiHa, CaSki) were purchased from the Shanghai Institute of Life Sciences Cell Resource Center, Shanghai, China. All cell lines were cultured in DMEM medium (Gibco, USA) supplemented with 10% fetal bovine serum (FBS) and 1% penicillin/streptomycin (Biowest, France). Normal cervical tissues were obtained from premenopausal women who underwent hysterectomy because of myoma or adenomyoma at the Department of Obstetrics and Gynaecology at Shanghai Changzheng Hospital. Primary cervical epithelial cells were digested from tissues by DispaseII (Roche, Switzerland) and Trypsin-EDTA Solution (Biowest, France) and were maintained in Keratinocyte-SFM (Gibco, USA). All cell cultures were maintain at 37°C in a 5% CO_2_, humidified incubator.

### Quantitative real-time PCR analysis

Total RNA was extracted from frozen tumor specimens and cell lines using Trizol reagent (Invitrogen, USA) and reverse-transcribed using random primers and an M-MLV Reverse Transcriptase Kit (Invitrogen, USA) according to the manufacturer's instructions. The expression of filtered lncRNAs and associated encoding genes was measured by TaqMan probe quantitative real-time PCR (qPCR) using Premix Ex Taq (TakaraBio, Japan) on an Applied Biosystems StepOne Real Time PCR system (Applied Biosystems, USA) according to manufacturer's instructions. H18S was used as an internal standard, and each sample was analyzed in triplicate. Relative gene expression (fold change) was calculated using the 2^−△△Ct^ method. The probes and corresponding primers in this study were designed and synthesized by GenePharma(Shanghai, China). The sequences of primers and probes in qPCR are listed in Table S2. The primers of U6 were designed and synthesized by RiboBio (GuangZhou, China).The sequences of primers are not provided by the corporation.

### RNA immunoprecipitation

Nuclear and Cytoplasmic Protein Extraction Kit (Beyotime, China) combined with RNA-Binding Protein Immunoprecipitation Kit (Millipore, USA) were used in performing RIP experiment according to the manufacturer's instructions. The EZH2 antibody used for RIP are D2C9 (Cell Signaling Technology, USA). Co-precipitated RNAs were detected by reverse-transcription PCR (RT-PCR), agarose gel electrophoresis (AGE) and qPCR. Total RNAs (input control) and controls were also assayed to demonstrate that the detected signals were from RNAs specifically binding to EZH2. The gene-specific primers used in RIP experiment are presented in Table S2.

### siRNA transfection

HeLa and SiHa cells were plated in a 6-well plate in antibiotic-free growth medium supplemented with 10% FBS and cultured until 50–70% confluent. SiRNAs were mixed with Lipofectamine 2000 (Invitrogen, USA) in reduced serum medium (Opti-MEM, Gibco, USA) according to the manufacturer's instructions. Transfection was carried out for 48 h, followed by harvesting of treated cells for further studies. siRNAs were designed and synthesized by GenePharma (Shanghai, China). The siRNA sequences of lncRNA-EBIC, EZH2 and negative control used in this study are listed in Table S2.

### Wound healing assay

To perform the wound healing assay, cells were seeded on 6-well plates and transfected for 48 h with either lncRNA-EBIC siRNA or negative control siRNA, followed by the creation of an artificial, homogenous scratch wound on a confluent monolayer culture of HeLa and CaSki cells with a 200-µl pipette tip. Serum-free medium was added for a further 24 h of incubation, and the cells were imaged at 3 different time points (0, 12, and 36 h) using an inverted microscope. Percent of wound closure was calculated with Image J 1.47 software. Each experiment was performed in triplicate.

### Matrigel invasion assay

Matrigel invasion assays were performed in triplicate using Transwell^®^ permeable supports (Corning, USA) according to manufacturer's protocol. Briefly, cells were transfected with either lncRNA-EBIC siRNA or negative control siRNA for 48 h as described above, followed by plating onto a Matrigel-coated membrane in the upper chamber of a 24-well insert (8 µm pore size) containing serum free media. The bottom chamber contained DMEM media with 10% FBS. Cells were incubated at 37°C with 5% CO_2_ for 48 h after plating, after which the bottom of the chamber insert was fixed with methanol and stained with crystal violet. Cells that remained in the upper chamber were removed with a cotton swab. The number of cells that invaded through the membrane was determined from digital images captured on an inverted microscope and calculated with Image J 1.47 software.

### Western blot analysis

Cells were harvested in RIPA lysis buffer (Beyotime, China). Equal amounts of protein were separated by SDS-PAGE and transferred onto polyvinylidene fluoride membranes (Millipore, USA). The membranes were blocked in phosphate-buffered saline/Tween-20 containing 5% non-fat milk and incubated with antibody for EZH2 (Cell Signaling Technology, USA) or β-actin (Santa Cruz biotechnology). Then, the membranes were incubated with HRP-labeled IgG (KPL, USA) and detected using an Epson Perfection V300 Photo Scanner (Epson, Japan). Quantitative analysis was performed using AlphaEase FC software (Alpha Innotech, USA). Protein levels were normalized to β-actin.

### Statistical analysis

Statistical analyses were performed using SPSS version 18.0 software (SPSS, Inc., Chicago, IL)and GraphPad Prism 5.0 software. Numerical data were presented as means and standard errors. Differences between proportions were evaluated by the paired or unpaired Student's t-test. P values <0.05 were considered statistically significant.

## Results

### lncRNA and mRNA expression profiles in CC

Five CC and paired peritumoral tissues were analyzed for potential transcriptome changes in CC using an Affymetrix Glue Grant Human Transcriptome array. Hierarchical clustering showed systematic variations in the expression of lncRNAs and mRNAs between CC and paired peritumoral tissues. Compared with paired peritumoral tissues, 708 probe sets of lncRNAs increased and 836 probe sets decreased in CC tissues (Figure 1A), while 1288 mRNA differential probe sets increased and 901 mRNA probe sets decreased (Figure 1B).

**Figure 1:** lncRNA and mRNA expression profiles of cervical cancer (CC). Using heat map hierarchical clustering analysis, we identified 1544 lncRNAs (A) and 2189 mRNAs (B) that were differentially expressed in CC tissues but not in the paired peritumoral tissues (c, cancer tissue; p, peritumoral tissues; P<0.05). Up-regulation or down-regulation is represented as red or green, respectively.

### Gene co-expression network and candidate lncRNAs

An RVM t-test was used to identify the number of differentially expressed lncRNAs and mRNAs from microarray analysis of CC and paired peritumoral tissues. To filter the data, we first overlapped differential expression mRNAs with the Cervical Cancer Gene Database (CCDB.) We determined 12 down-regulated and 48 up-regulated mRNAs (Table S3), including APOD, ESR1, MMP1, PCNA, and EZH2, etc. Co-expression network analysis was performed between the 60 filtered mRNAs and 1545 differentially expressed lncRNAs. The network structure of the CC (Figure 2A) and peritumoral (Figure 2B) tissue samples was markedly different, implyapp:addword:implying that the co-expression patterns of mRNA and lncRNAs between CC and paired peritumoral tissues are different. Recent studies have demonstrated that the oncoproteins E7 of high-risk HPV16 could active the expression of EZH2 at transcriptional level which contributed to the proliferation and apoptotic resistance of CC cells [23]. Moreover, EZH2 are over-expressed in CC tissues and its high expression significantly correlates with aggressiveness [24]. More recently, studies have suggested that deregulated lncRNAs may have a general role in inducing genome-wide re-targeting of PRC2 which will result in aberrant expression of genes, ultimately lead to cancer or other diseases [11], [18]. Thus, we chose EZH2, a core subunit of the PRC2, for detection of potential lncRNAs involved in CC because it presented as a hub node with high degree centrality. Eleven mRNAs and nine lncRNAs (TI17313, TI13831, TI10124, TI18382, TI21327, TI18318, TI22687, TI09485, and ASK00420; (Table S4) that tightly interacted with EZH2 (interaction ≥0.865) were chosen from the EZH2 subnetwork in the co-expression network of the peritumoral group.

**Figure 2:** lncRNA-mRNA co-expression network. A display of the lncRNA-mRNA network for the 60 filtered mRNAs and 1545 differentially expressed lncRNAs in CC (A) and paired peritumoral tissues (B) is shown. Up-regulated RNAs are shown in red, and down-regulated RNAs are presented in blue. Nodes with a green ring represent lncRNAs. Nodes without a green ring represent mRNA. Node size represents the degree centrality.

### Validation of the candidate lncRNAs in CC tissues and cell lines

To validate the microarray data, we first analyzed TI17313, TI13831, TI10124, TI18382, TI21327, TI18318, TI22687, TI09485, and ASK00420 expression in 23 paired CC and peritumoral samples using qRT-PCR. Results showed that the expression of these lncRNAs was either increased or decreased in CC tissues as compared to paired peritumoral tissues (Figure 3A) and was consistent with the microarray results. LncRNA expression was then analyzed in CC cells and normal, primary cervical epithelial cells in the same manner. The levels of TI17313, TI13831, TI10124, and TI18318 were increased in 3 cancer cell lines (HeLa, SiHa, and CaSki) when compared with normal, primary cervical epithelial cells (Figure 3B). Expression of the 5 other lncRNAs was below the level of detection in cultured cells (data not shown). Taking into account the expression and difference of candidate lncRNAs in tissues and cells, we selected TI17313, TI13831, TI10124, and TI18318 for further study.

**Figure 3:** Validation of microarray data for tissue and cells by real-time RT-PCR (qRT-PCR). Nine candidate lncRNAs were validated in 23 paired CC and peritumoral tissue samples using qRT-PCR (A). Expression levels of TI17313, TI13831, TI10124, and TI18318 in CC cell lines relative to the levels in normal, primary cervical epithelial cells (B) are shown. *P<0.05, **P<0.01.

### lncRNA-TI17313 was associated with EZH2

To investigate whether there is a physical interaction between the four candidate lncRNAs and EZH2, RIP was performed using an EZH2 antibody and nuclear extracts of HeLa and SiHa cells. We observed that only TI17313 enriched significantly with the EZH2 antibody compared with IgG (control antibody) (Figure 4A, 4B), and there was no enrichment ofβ-actin and TI13831 (control RNA) (Figure 4C). Furthermore, to determine the intracellular localization of TI17313, we separated cytoplasmic and nuclear RNA of HeLa cells by Cytoplasmic & Nuclear RNA Purification Kit (Norgen Biotek, Canada) effectively. Then, RT-PCR and AGE showed that the transcript of TI17313 was mainly located in nucleus of CC cells (Figure S1). These data suggested an association between TI17313 and EZH2; therefore, we termed TI17313 as EZH2-binding lncRNA in cervical cancer (lncRNA-EBIC).

**Figure 4:** lncRNA TI17313 associates with EZH2. (A, B) RIP experiments were performed in SiHa and HeLa cells using the EZH2 antibody (Ab) to immunoprecipitate and specific primers to detect TI17313, TI13831, TI10124, and TI18318 respectively, and relative enrichments are shown. *P<0.05. (C) RIP experiments were performed using the EZH2 antibody (Ab) to immunoprecipitate a primer to detect β-actin and TI13831.

### lncRNA-EBIC silencing impaired CC cell migration and invasion in vitro

To evaluate the effects of lncRNA-EBIC on cellular behavior, CC cell lines were treated with siRNA to silence lncRNA-EBIC signaling. lncRNA-EBIC levels were significantly decreased in HeLa and SiHa cells treated with siRNA (Figure 5A). Cell-Counting Kit-8 assays and Annexin V-FITC flow cytometry analysis were performed, and cell proliferation and apoptosis were not obviously affected by down-regulation of lncRNA-EBIC (data not shown). A wound healing migration assay determined that siRNA-mediated lncRNA-EBIC silencing impaired CC cell migration *in vitro* (Figure 5B). A Matrigel invasion assay showed decreased invasion through matrigel in lncRNA-EBIC silenced cells as compared with control (Figure 5C). These data suggest that lncRNA-EBIC positively regulates the migration and invasion of CC cells.

**Figure 5:** Silencing of lncRNA-EBIC by siRNA decreases motility and invasion of CC cells. LncRNA-EBIC levels were significantly decreased in HeLa and SiHa cells treated with lncRNA-EBIC siRNA (A). Wound healing (B) and Matrigel invasion assays (C) indicated that the motility and invasion of HeLa and SiHa cells were impaired by treatment with lncRNA-EBIC siRNA compared with mock and negative control. Cellular profiles are representative of 3 independent experiments. Statistical analyses are shown as right panels respectively. *P<0.05.

### lncRNA-EBIC associated with EZH2 repressed the expression of E-cadherin

Disruption of cell-cell adhesion and down-regulated E-cadherin are the initial stages of tumor invasion. Increasing evidence has shown that E-cadherin expression is repressed in cancer and reduced expression has been linked to metastasis. Furthermore, studies have demonstrated that EZH2 could mediate transcriptional silencing of E-cadherin by trimethylation of H3 lysine 27 [18], [25]. Thus, we speculated that the association between lncRNA-EBIC and EZH2 might subsequently result in a decrease of E-cadherin expression to promote CC cell invasion. To test it, we investigated the changes of E-cadherin mRNA and protein expression levels in lncRNA-EBIC siRNA transfected HeLa and SiHa cells. We found that lncRNA-EBIC siRNA treatment could increase the expression levels of E-cadherin in mRNA and protein, leaving EZH2 expression unchanged (Figure 6A, 6B). Next, EZH2 siRNA combined with lncRNA-EBIC or NC siRNA was used to transfect CC cells respectively, and we further observed that E-cadherin expression levels were also increased in both groups (Figure 6C). The effectiveness of EZH2 siRNA is presented in Figure S2. These data implied that lncRNA-EBIC could inhibit E-cadherin by associating with EZH2, and lncRNA-EBIC might act as a facilitator in recruiting EZH2 to the promoter region of E-cadherin. lncRNA-EBIC and EZH2 may be two interdependent components of the H3K27me3 process.

**Figure 6:** The expression levels of lncRNA-EBIC, EZH2 and E-cadherin mRNA were detected by qPCR after transfection of lncRNA-EBIC siRNA or negative control in HeLa and SiHa cells (A, B, left panel). Meanwhile, western blot analysis of EZH2 and E-cadherin were performed in CC cells treated with siRNA (A, B, right panel). Analysis of E-cadherin mRNA and protein levels were performed in CC cells treated with EZH2 siRNA+lncRNA-EBIC siRNA or EZH2 siRNA+negative control. *P<0.05.

## Discussion

Genome-wide transcriptome studies showed that nearly 10- to 20-fold more genomic sequence is transcribed to lncRNA than to protein-coding RNA. Finding new molecules and mechanisms could shed light on the complexity of various biological processes, including cellular development and human diseases [26], [27].

Increasing evidences in recent years showed that aberrant lncRNA expression is emerging as a major component of the cancer transcriptome. However, the overall pathophysiological contribution of lncRNAs to the initiation and progression of CC is still largely unknown. Recently, a rash of studies reveals that lncRNAs are important cis-/trans-regulators of gene activity, which means most lncRNAs may involve in the regulation of gene expression [28]. Thus, the co-expression network between lncRNAs and mRNAs is a significant approach to study the potential functions of lncRNAs. To explore the role of lncRNAs in cervical cancer, we first used a transcriptome microarray to evaluate lncRNA and mRNA expression profiles in CC and paired peritumoral tissues. Microarray combined with gene co-expression analysis revealed a set of differentially expressed lncRNAs and mRNAs.

EZH2, a core component of PCR2, is a pivotal enzyme in histone modification that plays a key role in catalyzing H3K27me3, resulting in transcriptional silencing of target genes [29]. For example, studies have suggested that EZH2 can inhibit E-cadherin expression through this methylation, thereby increasing cancer invasiveness and metastasis [4], [14]. However, relatively little is known about how EZH2 is recruited to target genes [30]. Recently, some studies have indicated that lncRNAs have the ability to recruit PRC2 to target loci in mammals via EZH2. For example, HOTAIR may induce PRC2 to localize with related promoters, leading to epigenetic silencing of metastasis suppressor genes in breast cancer [18]. For another example, lncRNA H19 could inhibit E-cadherin expression by transcriptional repression of the promoter through enrichment of EZH2 [17].

With regard to CC, some previous studies also showed that the over-expression of EZH2 is associated with aggressiveness and malignant progression of CC [23], [24]. As our microarray showed, the expression level of EZH2 was up-regulated in tumor tissues and presented as a hub node with high degree centrality. Thus, we chose EZH2 for detection of potential lncRNAs involved in CC. According to gene co-expression analysis, we determined 9 candidate lncRNAs which tightly interacted with EZH2.

In these candidate lncRNAs, we found that lncRNA-TI17313 expression levels were significantly increased in CC tissues and cell lines. TI17313 is a 1201bp in length noncoding RNA transcribed from a processed pseudogene located in chromosome 16q and coded RP11-144N1.1 (Ensembl version ENSG00000262904). Like with most lncRNAs, TI17313 also shows lower conservation among species. Its sequence only conserves among the primates (http://asia.ensembl.org/Homo_sapiens/Location/Compara_Alignments?align = 654&db = vega&g = OTTHUMG00000177355&r = 16%3A74701404-74702604&t = OTTHUMT00000436401). Furthermore, we investigated the function and mechanisms of this candidate lncRNA. RIP showed a physical interaction of lncRNA-TI17313 with EZH2; therefore, we named lncRNA-TI17313 as lncRNA-EBIC. Subsequently, loss-of-fuction assays showed that decreased expression of lncRNA-EBIC inhibited CC cell migration and invasion in vitro. These studies suggested that lncRNA-EBIC might act as a oncogene through cooperating with EZH2. Meanwhile, the association of lncRNA-EBIC with EZH2 also provided a hint to the complicated regulation mechanism of EZH2.

Tumor migration and invasion are the major catalysts of morbidity and mortality in cancer patients. E-cadherin is a tumor suppressor gene that plays a critical role in the malignant progression of epithelial tumors and inhibits epithelial to mesenchymal transition [31]. CC frequently presents with decreased expression of E-cadherin and is associated with the HPV oncoproteins E6 and E7 [32]. Over-expression of EZH2 has been reported to decrease the level of E-cadherin gene expression through H3K27me3 in the E-cadherin promoter [4], [14]. In our study, we found that down-regulation of lncRNA-EBIC could increase the expression levels of E-cadherin. Meanwhile, decreasing EZH2 expression level but leaving lncRNA-EBIC unchanged also could promote E-cadherin expression.

Because there are no explicit information about the transcription start/terminal sites and full-length sequence of lncRNA-EBIC, we are currently not available to perform the gain-of-function of lncRNA-EBIC and study the potential mechanism in more detail. However, the association of lncRNA-EBIC with EZH2 suggested a role of lncRNA-EBIC in the epigenetic control of gene expression. More important, in this research, we first revealed the differencially expressed lncRNAs in CC. Among these candidate lncRNAs, we demonstrated that an up-regulated lncRNA in CC tissues and cells was associated with EZH2, termed lncRNA-EBIC. lncRNA-EBIC could promote CC cells invasion by associating with EZH2 and subsequently repressing E-cadherin expression, suggesting that lncRNA-EBIC might act as a facilitator in recruiting EZH2 to target genes. Thus, our results suggest an important role for epigenetic mechanisms in cervical CC pathogenesis. A better understanding of the role of lncRNAs in modulating the epigenetic activity will provide more targets for anticancer therapy, and therefore is promising for the individualized treatment of cervical cancer patients.

## Supporting Information

Figure S1 **To determine the intracellular localization of lncRNA-EBIC, Cytoplasmic & Nuclear RNA Purification Kit (Norgen Biotek, Canada) was used to separate cytoplasmic and nuclear RNA of HeLa cells.** Then, RT-PCR and AGE showed that the transcript of lncRNA-EBIC was mainly located in nucleus of CC cells.
(TIF)

Figure S2 **Analysis of EZH2 mRNA and protein levels were performed in HeLa and SiHa cells treated with EZH2 siRNA.** *P<0.05.
(TIF)

Table S1 The data of cervical cancer specimens in this project.
(DOC)

Table S2 Oligonucleotide Sequences used in this study.
(DOC)

Table S3 The 60 differential mRNAs screened out from the overlap outcome of microarray data and CCDB.
(DOC)

Table S4 The node information of EZH2 sub-network in the coexpression network of para-tumor group.
(DOC)

## References

[1] JemalA, BrayF, CenterMM, FerlayJ, WardE, et al (2011) Global cancer statistics. CA Cancer J Clin 61: 69–90.2129685510.3322/caac.20107

[2] ChangSC, WooJS, YauV, GorzalkaBB, BrottoLA (2013) Cervical cancer screening and chinese women:insights from focus groups. Front Psychol 4: 48.2342354710.3389/fpsyg.2013.00048PMC3573354

[3] KriegerN, BassettMT, GomezSL (2012) Breast and cervical cancer in 187 countries between 1980 and 2010. Lancet 379: 1391–1392.2250087610.1016/S0140-6736(12)60596-0

[4] EggerG, LiangG, AparicioA, JonesPA (2004) Epigenetics in human disease and prospects for epigenetic therapy. Nature 429: 457–463.1516407110.1038/nature02625

[5] JonesPA, BaylinSB (2002) The fundamental role of epigenetic events in cancer. Nat Rev Genet 3: 415–428.1204276910.1038/nrg816

[6] KrolJ, LoedigeI, FilipowiczW (2010) The widespread regulation of micro-RNA biogenesis,function and decay. Nat Rev Genet 11: 597–610.2066125510.1038/nrg2843

[7] QinW, DongP, MaC (2012) MicroRNA-133b is a key promoter of cervical carcinoma development through the activation of the ERK and AKT1 pathways. Oncogene 31: 4067–75.2217982910.1038/onc.2011.561

[8] HuarteM, RinnJL (2010) Large non-coding RNAs: missing links in cancer? Hum Mol Genet 19: R152–161.2072929710.1093/hmg/ddq353PMC2953740

[9] YangF, ZhangL, HuoXS, YuanJH, XuD, et al (2011) Long noncoding RNA high expression in hepatocellular carcinoma facilitates tumor growth through enhancer of zeste homolog 2 in humans. Hepatology 54: 1679–1689.2176990410.1002/hep.24563

[10] GibbEA, Becker-SantosDD, EnfieldKS, GuillaudM, NiekerkDv, et al (2012) Aberrant expression of long noncoding RNAs in cervical intraepithelial neoplasia. Int J Gynecol Cancer 22: 1557–1563.2309577410.1097/IGC.0b013e318272f2c9

[11] KhalilAM, GuttmanM, HuarteM, GarberM, RajA, et al (2009) Many human large intergenic noncoding RNAs associate with chromatin-modifying complexes and affect gene expression. Proc Natl Acad. Sci. USA 106: 11667–11672.10.1073/pnas.0904715106PMC270485719571010

[12] SparmannA, van LohuizenM (2006) Polycomb silencers control cell fate, development and cancer. Nat Rev Cancer 6: 846–856.1706094410.1038/nrc1991

[13] Simon JA, Lange CA (2008) Roles of the EZH2 histone methyltransferase in cancer epigenetics. Mutant Res 647(1): , 21–29.10.1016/j.mrfmmm.2008.07.01018723033

[14] CaoQ, YuJ, DhanasekaranSM, KimJH, ManiRS, et al (2008) Repression of E-cadherin by the polycomb groupprotein EZH2 in cancer. Oncogene 27: 7274–7284.1880682610.1038/onc.2008.333PMC2690514

[15] Li H, Cai Q, Godwin AK, Zhang R (2010) Enhancer of zeste homolog 2 promotes the proliferation and invasion of epithelial ovarian cancer cells. Molecular Cancer Research, 8(12): , 1610–1618.10.1158/1541-7786.MCR-10-0398PMC305972721115743

[16] Lu C, Han HD, Mangala LS, Ali-Fehmi R, Newton CS, et al. (2010) Regulation of tumor angiogenesis by EZH2. Cancer cell, 18(2): , 185–197.10.1016/j.ccr.2010.06.016PMC292365320708159

[17] LuoM, LiZ, WangW, ZengY, LiuZ, et al (2013) Long non-coding RNA H19 increases bladder cancer metastasis by associating with EZH2 and inhibiting E-cadherin expression. Cancer Letters 333: 213–221.2335459110.1016/j.canlet.2013.01.033

[18] GuptaRA, ShahN, WangKC, KimJ, HorlingsHM, et al (2010) Long noncoding RNA HOTAIR reprograms chromatin state to promote cancer metastasis. Nature 464: 1071–1076.2039356610.1038/nature08975PMC3049919

[19] WrightGW, SimonRM (2003) A random variance model for detection of differential gene expression in small microarray experiments. Bioinformatics 19: 2448–2455.1466823010.1093/bioinformatics/btg345

[20] YangH, CrawfordN, LukesL, FinneyR, LancasterM, et al (2005) Metastasis predictive signature profiles pre-exist in normal tissues. Clin Exp Metastasis 22: 593–603.1647503010.1007/s10585-005-6244-6PMC2048974

[21] PujanaMA, HanJD, StaritaLM, StevensKN, TewariM, et al (2007) Network modeling links breast cancer susceptibility and centrosome dysfunction. Nat Genet 39: 1338–1349.1792201410.1038/ng.2007.2

[22] Zhang B, Horvath S (2005) A general framework for weighted gene co-expression network analysis. Stat Appl Genet Mol Biol.; 4: :Article 17.10.2202/1544-6115.112816646834

[23] Holland D, Hoppe-Seyler K, Schuller B, Lohrey C, Maroldt J, et al. (2008) Activation of the enhancer of zeste homologue 2 gene by the human papillomavirus E7 oncoprotein. Cancer research, 68(23): , 9964–9972.10.1158/0008-5472.CAN-08-113419047178

[24] Fang J, Zhang M, Li Q (2011) Enhancer of zeste homolog 2 expression is associated with tumor cell proliferation and invasion in cervical cancer. The American journal of the medical sciences, 342(3): , 198–204.10.1097/MAJ.0b013e31821335a921629038

[25] Wang C, Liu X, Chen Z, Huang H, Jin Y, et al. (2013) Polycomb group protein EZH2-mediated E-cadherin repression promotes metastasis of oral tongue squamous cell carcinoma. Molecular carcinogenesis, 52(3): , 229–236.10.1002/mc.21848PMC340071322161744

[26] MercerTR, DingerME, MattickJS (2009) Long non-coding RNAs: insights into functions. Nat Rev Genet 10: 155–159.1918892210.1038/nrg2521

[27] WiluszJE, SunwooH, SpectorDL (2009) Long noncoding RNAs: functional surprises from the RNA world. Genes Dev 23: 1494–1504.1957117910.1101/gad.1800909PMC3152381

[28] Nagano T, Fraser P (2011) No-nonsense functions for long noncoding RNAs. Cell, 145(2): , 178–181.10.1016/j.cell.2011.03.01421496640

[29] CaoR, ZhangY (2004) The functions of E(Z)/Ezh2-mediated methylation of lysine 27 in histone H3.Curr Opin Genet Dev. 14: 155–164.10.1016/j.gde.2004.02.00115196462

[30] SimonJA, LangeCA (2008) Roles of the EZH2 histone methyltransferase in cancer epigenetics. Mutat Res 647: 21–29.1872303310.1016/j.mrfmmm.2008.07.010

[31] LarueL, BellacosaA (2005) Epithelial-mesenchymal transition in development and cancer: role of phosphatidylinositol 3′ kinase/AKT pathways. Oncogene 24: 7443–7454.1628829110.1038/sj.onc.1209091

[32] D'CostaZJ, JollyC, AndrophyEJ, MercerA, MatthewsCM, et al (2012) Transcriptional repression of E-cadherin by human papillomavirus type 16 E6. PLOS One 7: e48954.2318913710.1371/journal.pone.0048954PMC3506579

